This article has been retracted.

# Establishment of Criteria for Molecular Differential Diagnosis of MPLC and IPM

**DOI:** 10.3389/fonc.2020.614430

**Published:** 2021-01-21

**Authors:** Xiaohui Wang, Yuan Gong, Jianfei Yao, Yan Chen, Yuemin Li, Zhen Zeng, Yinying Lu, Lele Song

**Affiliations:** ^1^Department of Oncology, The Fifth Medical Center of the Chinese People's Liberation Army (PLA) General Hospital, Beijing, China; ^2^The Medical Division, HaploX Biotechnology, Shenzhen, China; ^3^Department of Gastroenterology, The Second Medical Center of the Chinese PLA General Hospital, Beijing, China; ^4^Department of Radiotherapy, The Eighth Medical Center of the Chinese PLA General Hospital, Beijing, China

**Keywords:** non-small cell lung cancer (NSCLC), multiple primary lung cancer (MPLC), intrapulmonary metastasis (IPM), next-generation sequencing (NGS), epidermal growth factor receptor (EGFR), driver gene

## Abstract

**Backgrounds:**

Differential diagnosis of multiple primary lung cancer (MPLC) and intrapulmonary metastasis (IPM) is one difficulty in lung cancer diagnosis, and crucial for establishment of treatment strategies and prognosis prediction. This study aims to establish the criteria for molecular differential diagnosis of synchronous MPLC and IPM by the next-generation sequencing (NGS) method.

**Methods:**

Training cohort included 30 synchronous MPLC (67 samples) patients and 5 synchronous IPM (13 samples) patients with adenocarcinoma. Criteria of MPLC/IPM differential diagnosis were established by results from a NGS-based 605-gene panel test. Subsequently, 16 patients (36 samples) were recruited as the validation cohort to verify the criteria.

**Results:**

IPM lesions showed a high degree of mutation overlap with an average concordance rate of 60.2% (range: 15.8%–91.7%). IPM lesions had at least three common alterations, including both high-frequency driver gene alterations and low-frequency gene alterations. In contrast, the average concordance rate of MPLC was 11.0% (range: 0.0%–100.0%), among which 66.7% (20/30) of patients had no common alterations (concordance rate: 0%). In the remaining 10 patients, 9 had only one overlapping alteration while 1 had two overlapping alterations, in which 6 patients had EGFR L858R overlapping mutation. Alterations were classified into trunk, shared, and branch subtypes. Branch alterations accounted for 94.4% of mutations in MPLC, while accounted for only 45.0% in IMP. In contrast, the ratio of trunk (38.3%) and shared (16.7%) alterations in IPM was significantly higher. The criteria for differentiating MPLC from IPM using 605-gene panel was established: 1) MPLC can be interpreted if no overlapping alterations is found; 2) MPLC is recommended if one overlapping high-frequency drive gene alteration and/or one overlapping low-frequency gene alteration are/is found; 3) IPM can be interpreted if more than three common alterations are found. Subsequently, 16 patients were recruited as the validation cohort in the single-blind manner to verify the criteria, and 14 MPLC and 2 IPM were identified, which was 100% consistent with the results from independent imaging and pathological diagnosis.

**Conclusions:**

NGS detection can distinguish synchronous MPLC from IPM and is a useful tool to assist differential diagnosis.

## Introduction

Lung cancer is one of the most common malignant tumors and is the leading cause of cancer-related death worldwide (1). The application of low-dose CT facilitated the detection of small lung nodules and early identification of high-risk lung cancer population (2). Due to the improvement of early detection methods, diagnosis and treatment of patients with multiple nodules has become a major challenge. One large retrospective cohort reported that 14.5% (559/3846) of NLCLC patients carried multiple lesions, in which 175 had synchronous tumors and 384 had metachronous tumors (3). Since the treatment strategy and prognosis for multiple primary lung cancer (MPLC) and intrapulmonary metastasis (IPM) are distinct from each other, differential diagnosis is necessary, which remains challenging in clinical practice.

The widely used criteria for clinical identification of MPLC and IPM were proposed by Martini and Melamed in 1975 (4). The diagnostic criteria were mainly based on the histological characteristics of tumors and had a strong practical value, but it was rather empirical without consideration of the biological and/or molecular features of tumors. More recently, the eighth edition of IASLC lung cancer TNM classification has described four patterns of presentation associated with multiple pulmonary sites of lung cancer, and recommended multidisciplinary diagnosis involving imaging, pathological and genomic diagnosis to discriminate MPLC from IPM (5). Previous studies have reported that MPLC and IPM can be identified by genetic analysis of tumor (6–8). For example, Schneider et al. conducted a comprehensive genetic test on 42 cases of multiple lung adenocarcinoma and found that 56% of the patients had genetic heterogeneity of each lesion (9). Study by Chen et al. also showed that most tumors had highly inconsistent mutations between independent primary sites (89.7%) (10). Although these studies supported the use of next-generation sequencing (NGS) panel to supplement imaging and histological examinations for robust identification of NSCLC clonal relationship, the use of NGS technology to distinguish MPLC from IPM remains challenging, since the boundary of MPLC and IPM is sometimes vague, especially for multiple lesions with identical pathological types. To this end, we established training and validation cohorts with patients with synchronous multiple adenocarcinoma lesions, and conducted targeted sequencing containing 605 cancer-related genes. We proposed and validated clear criteria for distinguishing MPLC from IPM, which is helpful for future differential diagnosis.

## Methods and Materials

### Ethics Approval and Consent to Participate

All experiment plans and protocols for the study were submitted to the ethics/licensing committee of the participating hospitals for review and approval before the start of the clinical study and were approved by the corresponding committee of the hospital. No informed consent was required as this study used retrospective samples for testing, while patients were informed of the test results. All experiments, methods, procedures, and personnel training were carried out in accordance with relevant guidelines and regulations of the participating hospitals and laboratory.

### Study Design, Patients, and Samples

The cohort study was a retrospective study designed and implemented to include as many MPLC and IPM adenocarcinoma patients as possible, as long as the tissue samples were available for NGS (**Table 1**). The main inclusion criteria included adults over 18 years old and those have complete clinicopathological information and confirmed diagnosis of lung adenocarcinoma by imaging examination (including endoscopy, ultrasound, MRI, CT, etc.) and subsequent pathological examination. Multiple cancer lesion samples must be available for NGS tests. The main exclusion criteria included those with suspected lung metastasis of cancers other than lung, and those with no tissue samples or control samples available. Patients with incomplete information were also excluded. As a result, a total of 51 patients with complete sample and clinical information were included with confirmed imaging and pathological diagnosis, including 44 MPLC and 7 IPM. The training and validation cohort were established in roughly 2:1 ratio. 35 patients were included in the training cohort and the rest 16 were included in the validation cohort. Samples for both training and validation cohorts were collected retrospectively. The validation cohort was tested in single-blind manner, in which the investigators for NGS tests and data interpretation and result interpretation were blinded to imaging and pathological diagnosis. Determination of MPLC or IPM by clinicians before any genetic tests followed the IASLC guideline on the classification of lung cancers with multiple pulmonary sites of involvement (4, 5). In brief, the discrimination of MPLC and IPM was based on the test results of imaging examination (CT scanning identifying imaging features), the findings during surgery (anatomical evidence of separate or metastatic lesions), the results of pathological examination on resected lymph nodes (evidence of nodal metastasis), and the histological examination of primary tumors and the surgical margin (histological subtypes of primary tumors). Two pathologists examined all biopsies independently and consensus was reached for all samples. Doctors made an interpretation on whether the tumors were synchronous primary lesions or primary tumor with metastasis based on the outcomes of the all available evidence. The cancer stage was based on natural distribution of all available cancer patients, including 30 stage I, 10 stage II, 5 stage III, and 6 stage IV patients (**Table 1**). Clinical status of patients was determined before the collection of samples [formalin-fix paraffin-embedded (FFPE) samples], and blood samples were available from all recruited subjects for genomic DNA control.

**Table 1:** Clinicopathological information for lung cancer patients involved in this study.

Clinicopathological factors			Overall	Training cohort	Validation cohort
Number of patients			51	35	16
Age, mean (range)			57.3 (34~78)	57.1 (34~78)	57.8 (40~69)
Gender					
	Male, n (%)		38	25 (71.4%)	13 (81.3%)
	Female, n (%)		13	10 (28.6%)	3 (18.7%)
Stage					
		I	30	21	9
		II	10	7	3
		III	5	3	2
		IV	6	4	2
Lesion type					
	MPLC, n (%)		44	30 (85.7%)	14 (87.5%)
	IPM, n (%)		7	5 (14.3%)	2 (12.5%)
Location of multiple nodules					
ipsilateral, same lobe			14	12 (34.3%)	2 (12.5%)
ipsilateral, different lobes			34	21 (60.0%)	13 (81.3%)
	bilateral		3	2 (5.7%)	1 (6.2%)

MPLC, multiple primary lung cancer; IPM, intrapulmonary metastasis.

### Sample Preparation, Targeted NGS, and Data Processing

For the FFPE samples, ten 5-μm tumor slices were used for DNA extraction using the QIAamp DNA FFPE Kit (QIAGEN, Valencia, CA, USA) following the manufacturer’s instructions. DNA from peripheral blood lymphocytes (PBLs) was extracted using the RelaxGene Blood DNA system (Tiangen Biotech Co., Ltd., Beijing, China) according to the manufacturer’s instructions. DNA was quantified with the Qubit 2.0 Fluorometer and the Qubit dsDNA HS assay kit (Thermo Fisher Scientific, Inc., Waltham, MA, USA) according to manufacturer’s instructions. In brief, fragmented genomic DNA underwent end-repairing, A-tailing and ligation with indexed adapters sequentially, followed by size selection using Agencourt AMPure XP beads (Beckman Coulter Inc., Brea, CA, USA), and DNA fragments were used for library construction using the KAPA Library Preparation kit (Kapa Biosystems, Inc., Wilmington, MA, USA) according to the manufacturer’s protocol. Hybridization-based target enrichment was carried out with HaploX pan-cancer gene panel (605 cancer-relevant genes, HaploX Biotechnology, gene list was provided in **Supplementary Table 1**) and Pre−LM−PCR Oligos (Kapa Biosystems, Inc.) in 50-μl reactions, and seven to eight PCR cycles were performed depending on the amount of DNA input. DNA sequencing was then performed on the Illumina Novaseq 6000 system according to the manufacturer’s recommendations at an average depth of 5000× for tissue.

Sequencing data were de−multiplexed and aligned to the hg19 genome (GRch37) using Burrows−Wheeler Aligner (http://bio-bwa.sourceforge.net/) version 0.7.15−r1140 using default settings. Pileup files for properly paired reads with mapping quality ≥60 were generated using Samtools (http://www.htslib.org/). Somatic variants were determined using VarScan2 (http://varscan.sourceforge.net/). Allele frequencies were calculated for all Q30 bases. Using a custom Python script, previously identified tumor DNA mutations were intersected with a Samtools mpileup file generated for each sample, and the number and frequency were then calculated for each mutation. A mutation was identified if ≥5 mutant reads were identified and ≥1 mutant read was identified on each strand. Matched genomic DNA from white blood cells was used as control.

### Statistics, Data Analysis, Calculation of TMB, and Molecular Subtyping

Statistical analysis was performed and figures were plotted with Graphpad PRISM 5.0 software (GraphPad Software, Inc, La Jolla, CA 92037, USA). Student t-test was performed when two groups were compared, and ANOVA and *post hoc* tests (Bonferroni test) were performed when three or more groups were compared. Chi-square test and Fisher test were performed when rate or percentage was compared for significance. Keplan-Meier analysis was performed and survival curves were plotted with PRISM 5.0 software. Mutation spectrum figures were made with the R software (https://www.r-project.org/). “*”: P < 0.05; “**” P < 0.01; “***”: P < 0.001.

## Results

### Establishment of Criteria for Distinguishing MPLC From IPM

In order to study the diagnostic potential of differential molecular features in MPLC and IPM, we established a training cohort of 30 MPLC and 5 IPM, and thoroughly investigated the mutational alterations of all lesions. **Figure 1** shows the mutational spectrum of all lesions in MPLC and IPM, in which two to four lesions for each patient are shown. It can be observed that in 30 MPLC patients, 18/30 patients exhibited lesions at the same lung but different lobes (MPLC-SD), and 10 patients exhibited lesions at the same lung and same lobe (MPLC-SS), while 2 patients exhibited lesions at bilateral lungs (MPLC-D). The IPM patients all exhibited lesions at different lobes of the same (ipsilateral) lung. Mutational spectrum showed that EGFR, RBM10, BRAF, MDM2, TP53, MET, ALK KRAS, APC, and ERBB2 were genes with highest mutational frequency, and the majority of mutations were SNV mutations, while INDEL mutations of EGFR (mainly 19del), and CNV mutations of EGFR, MDM2 and TERT were also identified. This mutational spectrum exhibited no difference to reported mutational spectrum in Chinese NSCLC patients (11, 12).

**Figure 1:** The mutational landscape of all lesions from the training cohort, including 30 MPLC and 5 IPM patients. The top 50 mutated genes are shown as indicated. Different types of mutations are shown in different colors. MPLC-SD, lesions at the same lung but different lobes; MPLC-SS, lesions at the same lung and same lobe; MPLC-D, lesions at bilateral lungs.

The inter-lesion mutational status for each patient in MPLC and IPM was further investigated (**Figure 2A**). Mutations were categorized into three types, including trunk mutations, which were common mutations for all lesions, and shared mutations, which were common mutations of some but not all lesions (e.g., shared by two out of three lesions), and branch mutations, which were unique mutations from a certain lesion. **Figure 2A** shows the distribution of all three types of mutations in each of the 30 MPLC and 5 IPM. It can be observed that 20 out of 30 MPLC had no trunk or shared mutation, but only branch mutations, suggesting that 66.7% of MPLC had no common mutations at all. The rest 10 MPLC showed only one trunk mutation and/or one shared mutation, exhibiting a very low level of common mutations. In contrast, the number of trunk or shared mutations was substantially higher in IPM, suggesting a huge difference in mutation components (**Figure 2A**). Further analysis showed that 94.4% of mutations in MPLC were branch mutations, compared with only 45.0% in IPM, while more than half of the mutations were trunk (38.3%) or shared (16.7%) in IPM (**Figure 2B**). Moreover, IPM exhibited significantly higher level of overall mutations per sample (normalized number of mutations) than MPLC (P = 0.046), suggesting a higher mutational burden for metastatic lesions (**Figure 2B**).

**Figure 2:** Mutation status and concordance rate for lesions of the training cohort. Panel **(A)** The number of mutations for all lesions of all patients with MPLC or IPM. Trunk, shared, and branch mutations are shown as indicated. Panel **(B)** Comparison of the normalized number of mutations (total number of mutations/number of patients) for MPLC and IPM. The ratio of trunk, shared, and branch mutations are shown as indicated. Panel **(C)** The concordance rate for each patient, with key common driver genes labeled. MPLC-SD, lesions at the same lung but different lobes; MPLC-SS, lesions at the same lung and same lobe; MPLC-D, lesions at bilateral lungs.

The concordance rate among multiple lesions for each patient in MPLC and IPM was studied in detail (**Figure 2C** and **Supplementary Figure 1**). IPM lesions showed an average concordance rate of 60.2% (range: 15.8%–91.7%), compared with 11.0% (range: 0.0%–100.0%) in MPLC. The concordance rate for the 20 MPLC with only branch mutations was 0%, while it varied from 5.3% to 100% for the rest 10 MPLC with trunk or shared mutations. Interesting, it was found that the trunk or shared mutations in MPLC were mostly high-frequency driver gene mutations, including those targeted by tyrosine kinase inhibitors (TKIs). Specifically, 6 out of the 10 MPLC patients showed trunk mutations of EGFR L858R, while the rest four showed KRAS G12C (shared), TERM amplification (trunk), DICER K1844N (trunk), and TNFRSF R228K (shared), respectively (**Figure 2C** and **Supplementary Figure 1A**). Apart from patient DP024, who showed both trunk EGFR L858R and shared ALK D1311N, the other nine MPLC patients all showed only one trunk or shared mutation. In contrast, the five IPM patients showed at least three trunk or shared mutations, including both high-frequency driver gene mutations and low-frequency mutations (**Figure 2C** and **Supplementary Figure 1B**).

Based on the above observations, we developed our interpretation criteria as a flowchart for discriminating MPLC from IPM (**Figure 3**). All lesions with available samples should be tested with the 605-panel test first, and the mutational landscape is compared for concordance rate and the number of overlapping mutations. If no common mutations are found among the lesions (concordance rate = 0%), MPLC can be interpreted. If the concordance rate is not 0%, the mutational status should be categorized into the following three conditions: Firstly, if TKI-related driver gene alterations, including EGFR (SNV, INDEL, Amp), ALK (fusion), ROS1 (fusion), MET (fusion, skipping, Amp), RET (fusion, Amp), BRAF (SNV, INDEL), and KRAS (SNV, INDEL) is found as the only common alteration, interpretation of MPLC is recommended; Secondly, if only one non-TKI–related gene alteration is found, or one TKI-related and one non-TKI–related gene alterations are found (total number of common mutations ≤ 2), lesions can be interpreted as MPLC; Thirdly, if more than three gene alterations are found, interpretation of IPM is recommended.

**Figure 3:** Flowchart shows the interpretation procedure and criteria for distinguishing MPLC from IPM. *TKI-related driver gene alterations include EGFR (SNV, INDEL, Amp), ALK (fusion), ROS1 (fusion), MET (fusion, skipping, Amp), RET (fusion, Amp), BRAF (SNV, INDEL), and KRAS (SNV, INDEL).

### Validation of Interpretation Criteria in Distinguishing MPLC From IPM

In order to validate the above criteria and rationalize the flowchart for discriminating MPLC from IPM, we collected samples from another 16 patients as the validation cohort (**Figures 4** and **5** and **Supplementary Figure 2**). Single blind study was performed with the samples, and the mutational landscape and interpretation results of MPLC and IPM were presented. As shown in **Figure 4**, EGFR, RMB10, CDK4, MDM2, TP53, CSMD3, TERT, and ERBB2 were genes with highest mutation frequency, which was similar to those in the training cohort. Two patients were interpreted as IPM (**Supplementary Figure 2B**) while the rest 14 appeared to be MPLC (**Supplementary Figure 2A**). This interpretation was supported by further analysis of mutational status and involved genes. **Figure 5A** shows that 11 patients (VP001-011) exhibited no common trunk or shared mutations among the lesions and their concordance rate was 0% (**Figure 5C**), and were interpreted as MPLC. Three patients (VP012-014) showed EGFR L858R or EGFR 19 del mutation as the only common mutation and therefore were also interpreted as MPLC (**Figures 5A, C**). Two patients (VP015-016) showed high concordance rate with more than three common mutations and therefore were interpreted as IPM (**Figures 5A, C**). The distribution of trunk, shared, and branch mutations showed similar pattern to the training cohort (**Figure 5B**). As a result, our interpretation was 100% consistent with the interpretation from independent imaging and pathological examinations. These results validated the interpretation criteria for distinguishing MPLC from IPM.

**Figure 4:** The mutational landscape of all lesions from the validation cohort, including 14 MPLC and 2 IPM patients. The top 50 mutated genes are shown as indicated. Different types of mutations are shown in different colors. MPLC-SD, lesions at the same lung but different lobes; MPLC-SS, lesions at the same lung and same lobe; MPLC-D, lesions at bilateral lungs.

**Figure 5:** Mutation status and concordance rate for lesions of the validation cohort. Panel **(A)** The number of mutations for all lesions of all patients with MPLC or IPM. Trunk, shared, and branch mutations are shown as indicated. Panel **(B)** Comparison of the normalized number of mutations (total number of mutations/number of patients) for MPLC and IPM. The ratio of trunk, shared, and branch mutations are shown as indicated. Panel **(C)** The concordance rate for each patient, with key common driver genes labeled. MPLC-SD, lesions at the same lung but different lobes; MPLC-SS, lesions at the same lung and same lobe; MPLC-D, lesions at bilateral lungs.

## Discussion

Differentiation between MPLC and IPM has always been a difficulty in clinical diagnosis of lung cancer with multiple lesions. The eighth edition of IASLC lung cancer TNM classification presented four patterns of disease that manifest multiple pulmonary sites of lung cancer (5). The patients in our study were all classified into adenocarcinoma and fell into the second and third types, i.e., separate tumor nodules or multifocal ground glass or lepidic (GG/L) nodules. The IASLC classification relied on imaging and pathological characteristics to make diagnosis, and provided evidence for staging to guide subsequent therapy, but did not provide clear distinguishing criteria between MPLC and IPM if separate nodules with the same pathological type are present. Therefore, there are still quite a few patients with multiple separate or GG/L nodules, who need confirmed diagnosis. Our study focused on adenocarcinoma and provided an easy and quick method for distinguishing MPLC from IPM using the NGS-based panel test.

We found that high heterogeneity was one major feature for MPLC, in which no or very few common alterations were found among primary multiple lesions. Separate lesions with no common mutations can be easily interpreted as MPLC, however, multiple lesions with common alterations need to be carefully examined and interpreted. Our study suggested that EGFR L858R was the most frequent common mutation for MPLC, and its presence without any other mutations indicated MPLC. Previous studies suggested that the prevalence of EGFR mutations in East Asian population was approximately 50% (13–15), in which EGFR L858R and EGFR 19del were the two most frequent mutations with roughly equal prevalence of around 20% in lung adenocarcinoma patients (13–15). Interestingly, we found in the training and validation cohorts that the prevalence of EGFR L858R far overweighed the prevalence of EGFR 19 del (eight patients with EGFR L858R versus one patient with EGFR 19del). Since the prevalence of EGFR L858R in our cohorts (8/51 = 15.7%) showed essentially no difference to the whole adenocarcinoma population, this observation suggested a negative selection for EGFR 19del mutations in MPLC. Moreover, the presence of other high frequency driver gene mutations, such as KRAS, TERT, and DICER1, suggested that a chance of common driver gene mutations existed in MPLC, which could be frequency-dependent. Since IPM in our cohorts all exhibited at least three common mutations and generally high concordance rate and high mutational burden, possibly due to comprehensive increase in the number of mutations, it can be concluded from our data that MPLC should be given priority in diagnosis for patients with only one common driver gene mutation among separate lesions, especially when multiple non-overlapping mutations are found. Latest evidence suggest that TKI-related EGFR mutations and KRAS G12D led to lower TMB compared with those without mutations (16, 17). In contrast, our own data suggest that lung cancer patients with TP53 mutations but without EGFR or KRAS mutations may have higher TMB than those without TP53 mutations. There is also evidence suggesting that mutations in Notch, Wnt, Hippo, PI3K, and Myc pathways may lead to higher TMB (16). Therefore, it appeared that the correlation between driver gene mutations and TMB can be categorized. Key TKI-related driver mutations may lead to lower TMB while pathway-related mutations may lead to higher TMB.

In this study, we categorized the alterations into trunk, shared, and branch types, and this allowed us to calculate the concordance rate among lesions for each patient. Branch alterations were the predominant type for MPLC while much higher trunk components were found with IPM. This reflected the clonal evolution among IPM lesions, in which trunk alterations were most likely clonal and shared or branch mutations were possibly subclonal (7, 18). Meanwhile, IPM appeared to have significantly higher total number of mutations than MPLC, suggesting an expansion of mutational clones during the spread of IPM. We also found that MPLC generally exhibited low concordance rate, except those with sole common driver gene mutations. In contrast, IPM generally exhibited much higher concordance rate, also reflecting the clonal properties of the disease. These observations suggested that the distinct molecular features of MPLC and IPM can be used to distinguish the two subtypes of multiple lung cancer, which is helpful for subsequent diagnosis and intervention.

MPLC and IPM and their differentiation have been investigated in previous studies. Several studies have reported that IPM exhibited high level of mutation concordance while the concordance for MPLC was much lower (3, 19, 20). Although concordance appeared to be statistically significant between MPLC and IPM in previous reports and the present study, it is not an applicable distinguishing indicator for individuals with MPLC or IPM, as some low-mutated MPLC lesions with common driver gene mutations may exhibit high concordance rate. Mutations of some driver genes, such as EGFR, KRAS, and TP53, were suggested to be useful as clonal markers in MPLC (20–23). However, only a limited number of gene mutations were analyzed in these reports, and discrimination between MPLC and IPM by driver genes alone remains difficult. It appeared that common mutations among MPLC lesions were due to coincidence of high-frequency driver gene mutations, while common mutations among IPM lesions were due to clonal expansion. There is so far no criteria on the number of genes that should be tested for distinguishing MPLC from IPM using the NGS method; however, it can be suggested from our study that the number should be large enough to cover both high and low frequency cancer-related genes, which involves consideration on both mutational frequency and diversity. This ensures enough alteration information for interpretation. The 605-gene panel used in this study was designed as a pan-cancer tool for detecting mutations in all solid tumors and therefore contained most lung cancer-related genes. Our study proved that this panel was large enough for mutation detection and had enough resolution in discriminating MPLC from IPM.

Although the method in our study provided good discrimination between MPLC and IPM in adenocarcinoma, diagnosis solely by NGS still have some limitations, and combination with imaging and pathological examinations is still necessary to ensure accurate diagnosis. Firstly, the number of patients in our cohorts was still limited, especially for IPM patients. The incidence for patients with separate lung cancer lesions was approximately 15% in all lung cancer patients (3), and it appeared from previous reports and our study that the majority of them were MPLC but not IPM; therefore, IPM seemed to be a more scarce subtype. More IPM cases and detailed comparison between MPLC and IPM are still needed to ensure the reliability of the established criteria of our study. Secondly, the diagnosis for some individuals with low number of mutations cannot be confirmed with NGS results alone. For example, separate lesions in patient DP024 had a common high-frequency EGFR L858R mutation and a common low-frequency ALK D1311N mutation, with an overall concordance rate of 33.3%. Diagnosis by NGS alone was still difficult for this patient, and combination diagnosis with CT and pathology is still necessary. Imaging test can provide unique evidence for MPLC and IPM distinguishment. A recent study established the algorithm for distinguishing MPLC from IPM by combining characteristics of lesions from CT/PET imaging and achieved good diagnostic efficacy (24). Thirdly, the criteria established in this study were based on the 605-gene panel. Whether the criteria are applicable for other NGS tests needs further validation. Fourthly, in this study, we focused on synchronous lung adenocarcinoma, whether the same principle can be applied to squamous cell carcinoma or small cell lung cancer is not known, and whether metachronous multiple lesions can be categorized using the same method is not known.

In clinical practice, it appeared that the majority of MPLC and IPM synchronous adenocarcinoma can be discriminated by NGS panel test, while a small proportion of patients appeared to be difficult in direct interpretation, which still needs the combination of imaging and pathological examinations. This was partly due to the difficulty in establishing definite criteria in genetic interpretation, because different NGS panels cover different number of genes and different genetic alterations, and the NGS test has not been normalized for MPLC and IPM differential diagnosis. To tackle this issue, we would try using whole-exome sequencing in future to obtain a full profile of mutational landscape of all lesions, as we found some patients had very limited number of mutations in NGS panel test, which complicated the interpretation. Furthermore, an algorithm combining imaging tests, pathological examinations and NGS test should be established to increase the confidence in MPLC and IPM differential diagnosis, which we believe will greatly enhance the accuracy in interpretation and could become a future routine clinical practice.

In conclusion, we found that NGS panel test was an effective tool for distinguishing lung MPLC from IPM. For those cases that cannot be distinguished by imaging and histopathology, the overlap rate and mutational status defined by NGS can be referred for diagnostic confirmation.

## Data Availability Statement

The original contributions presented in the study are publicly available. This data can be found here: https://bigd.big.ac.cn/bioproject/browse/PRJCA003895.

## Ethics Statement

The studies involving human participants were reviewed and approved by The Fifth Medical Center of the Chinese PLA General Hospital. The patients/participants provided their written informed consent to participate in this study.

## Author Contributions

LS, XW, ZZ, and YYL designed the study. YG, JY, YC, and YML recruited the subjects, collected the samples, and liaised with the laboratory. XW, YG, and LS analyzed the data. XW, YG, and LS made the figures and tables and wrote the manuscript. LS, ZZ, and YYL proofread the manuscript. LS submitted the manuscript. All authors contributed to the article and approved the submitted version.

## Funding

This study was supported by the Special Funds for Strategic Emerging Industry Development of Shenzhen (Grant Number 20170922151538732) and the Science and Technology Project of Shenzhen (Grant Number JSGG20180703164202084). This study was also supported by the National Science and Technology Major Project (2018ZX10302205-001), the National Key R&D Program of China (2017YFC0908401), and the National Science and Technology Major Project (2018ZX10723204 and 2018ZX10302205). This study was also supported by the Special health research projects of 2019 funded by the Chinese PLA general hospital (NLBJ-2019003). All funders did not participate in the study design, study implementation, data collection, data analysis, data interpretation, and manuscript writing of the study.

## Conflict of Interest

XW, LS, and JY are employees of HaploX Biotechnology.

The remaining authors declare that the research was conducted in the absence of any commercial or financial relationships that could be construed as a potential conflict of interest.

## Supplementary Material

Supplementary Figure 1 The mutational status for all lesions in all patients of the training cohort. Panels **(A, B)** show the mutational status for MPLC and IPM patients, respectively.

Supplementary Figure 2 The mutational status for all lesions in all patients of the validation cohort. Panels **(A, B)** show the mutational status for MPLC and IPM patients, respectively.
